# Risk factors for distant metastasis of patients with primary triple-negative breast cancer

**DOI:** 10.1042/BSR20190288

**Published:** 2019-06-04

**Authors:** Yi Yao, Yuxin Chu, Bin Xu, Qinyong Hu, Qibin Song

**Affiliations:** Cancer Center, Renmin Hospital of Wuhan University, Wuhan, China

**Keywords:** distant metastasis, risk factor, TNBC

## Abstract

**Objective:** Triple-negative breast cancer (TNBC) involves higher rates of recurrence and distant metastasis. The present study sought to characterize the risk factors for distant metastasis of TNBC.

**Methods:** The Surveillance, Epidemiology, and End Results (SEER) database was exploited to enroll patients diagnosed with TNBC from 2010 to 2015. The eligible patients were dichotomized into locoregional and distant metastasis at the time of diagnosis. Patients’ demographics and tumor features, and treatment were evaluated to identify the risk factors for distant metastasis of primary TNBC. The categorical variables were examined by chi-square tests. Univariate and multivariate logistic regression analyses were used to determine the risk factors for distant metastasis. Breast cancer-specific survival (BCSS) and overall survival (OS) were estimated by Kaplan–Meier plots with log-rank tests.

**Results:** We collected 26863 patients with primary TNBC, 1330 (5.0%) of them presented with distant metastasis. In the univariate analysis, all the variables indicated statistical significance. The significant variables were subsequently enlisted into the multivariate logistic regression analysis. Age > 50, higher clinical stage T and N, and tumor size > 5 cm were independent risk factors for distant metastasis of primary TNBC. Moreover, higher clinical stage T and stage N were independent risk factors for bone metastasis of the patients. TNBC patients with either bone or visceral metastasis have poor survival, with brain metastasis worst of all, though the OS difference was not statistically significant.

**Conclusions:** TNBC patients with larger age, higher clinical stage, larger tumor size were more predisposed to have distant metastasis. Great attention should be paid to the prognosis of these patients with distant metastasis.

## Introduction

Triple-negative breast cancer (TNBC) is a highly aggressive subtype of tumors that lack estrogen receptor (ER), progesterone receptor (PR) and human epidermal growth factor receptor 2 (HER2), which represents 15–20% of all breast cancers [1]. As the most lethal subtype of breast cancer, patients with TNBC have a high propensity for distant metastasis and limited treatment options, remaining a clinical challenge for oncologists [2]. Particularly, the TNBC was associated with a significantly poorer overall survival (OS) and prone to earlier recurrence and metastasis [3]. Considering the high risk of TNBC patients who are susceptible to develop distant metastasis, accurate breast cancer screening may help to reduce mortality by early detection of distant metastasis [4]. However, there is a relatively limited number of studies demonstrating reliable data on the relationship between traditional clinicopathological characteristics and metastatic pattern of TNBC. Most studies focus on metastatic tumors, neglecting adequate insight into cases without metastasis [5]. Moreover, the prognostic significance of distant metastasis pattern for TNBC patients at initial diagnosis has not been adequately evaluated. Studying the risk factors associated with distant metastasis of TNBC may contribute to the screening of patients at high risk and initiate early intervention.

The present study exploited the Surveillance, Epidemiology, and End Results (SEER) database to enroll a large population of TNBC cases for analysis. We investigated patients’ demographics (age, race, and marital status), tumor features (histologic type, grade, clinical stage T and N, tumor size), and treatment (surgery, chemotherapy, radiotherapy), in order to identify risk factors for distant metastasis of primary TNBC. The findings from the present study may lead to a deeper insight into the clinicopathological factors that will predict distant metastasis of TNBC prior to diagnosis. Our investigation will hopefully optimize the current evaluation of TNBC patients’ risk of distant metastasis at initial diagnosis and help make more suitable medical decisions.

## Methods

### Data source

All the data were acquired from the SEER 18 registries Research Data. We have submitted the data agreement form to the SEER administration.

The data released by the SEER database do not require informed patient consent because cancer is a reportable disease in every state of the United States.

### Patient selection

We used SEER*Stat version 8.3.5 to download data files directly. We used the following inclusion criteria to select eligible patients: (i) female breast cancer diagnosed from 2010 to 2015; (ii) unilateral breast cancer as the first and only cancer diagnosis; (iii) the breast cancer subtype was triple negative. (ii) The behavior recode for analysis was malignant. The diagnosis was not obtained from a death certificate or autopsy. We made a case table with information on the following variables: age at diagnosis, race recode, marital status, histologic type, grade, AJCC stage T and N, tumor size, surgery, chemotherapy, and radiotherapy. The patients with unknown data of these variables were excluded.

### Statistical analysis

Descriptive statistical analysis (chi-square test) was adopted to calculate the frequencies and proportion of patients presenting with localized/regional or distant metastatic TNBC according to the incorporated variables above. Univariate logistic regression analysis was used to preliminarily screen variables as potential risk factors related to distant metastasis. Subsequently, multivariate logistic regression analysis was utilized to adjust the confounding factors and verify the risk factors determined in the univariate analysis. For each variable, crude odds ratio (OR) and adjusted OR with 95% confidence interval (CI) were recorded in logistic regression analysis. The differences of breast cancer-specific survival (BCSS) and OS among each distant metastasis were analyzed by Kaplan–Meier plots with log-rank tests. All the statistical analysis were performed using SPSS statistical software, version 23.0 (SPSS, Chicago, IL, U.S.A.). A two-tailed *P*<0.05 was considered statistically significant.

## Results

### Patient selection

According to the aforementioned inclusion criteria, we preliminarily identified a total of 31942 women with primary TNBC from the SEER database. These patients had been diagnosed from 2010 to 2015. We subsequently excluded 5079 patients missing data of table variables. Ultimately, 26863 eligible patients were included in the present study.

### Patient and tumor characteristics

Among the included 26863 patients, 25533 women were locoregional, while the remainder 1330 patients (5.0%) had distant metastasis. The differences between locoregional and distant metastatic groups for all the variables indicated statistical significance (*P*<0.05) according to chi-square test. In the distant metastatic group, age 50–65 (42.0%), white race (68.0%), not married (55.7%), histologic type 8500 (82.2%), grade III (81.0%), stage T IV (41.0%), stage N1 (44.7%), tumor size > 5.0 cm (49.0%), no surgery (53.0%), chemotherapy (78.3%), and no radiotherapy (79.2%) are most remarkable. By contrast, more metastatic patients were age > 65 (32.1 vs 29.0%), black race (25.5 vs 20.2%), not married (55.7 vs 42.6%), other histologic type (14.1 vs 8.6%), grade IV (1.7 vs 0.8%), stage T III (19.2 vs 8.5%) and T IV (41.0 vs 4.6%), stage N3 (23.0 vs 3.9%), tumor size > 5 cm (49.0 vs 11.9%), no surgery (53.0 vs 4.0%), chemotherapy (78.3 vs 75.3%), and no radiotherapy (79.2 vs 50.0%). Furthermore, the risks for distant metastasis of primary TNBC seem to increase with age, grade, clinical stage T and N, and tumor size. Generally, the patients with higher age, black race, not married, other histologic type, higher grade, higher stage T and N, larger tumor size, no surgery, and no radiotherapy are more inclined to have distant metastasis. Further details of baseline data are available in Table 1.

**Table 1:** Demographics of TNBC patients dichotomized by distant metastasis (*n*=26863)

Characteristics	Total, *n* (%)	Locoregional, *n* (%)	Distant metastasis, *n* (%)	***P***-value
	*n*=26863	*n*=25533 (95.0)	*n*=1330 (5.0)	
**Age (years)**				<0.001
<35	1335 (5.0)	1271 (5.0)	64 (4.8)	
35–50	7099 (26.4)	6818 (26.7)	281 (21.1)	
50–65	10596 (39.4)	10038 (39.3)	558 (42.0)	
>65	7833 (29.2)	7406 (29.0)	427 (32.1)	
**Race**				<0.001
White	19316 (71.9)	18411 (72.1)	905 (68.0)	
Black	5505 (20.5)	5166 (20.2)	339 (25.5)	
Others	2042 (7.6)	1956 (7.7)	86 (6.5)	
**Marital status**				<0.001
Not married	11622 (43.3)	10881 (42.6)	741 (55.7)	
Married	15241 (56.7)	14652 (57.4)	589 (44.3)	
**Histologic type**				<0.001
8500	23020 (85.7)	21927 (85.9)	1093 (82.2)	
8523	764 (2.8)	747 (2.9)	17 (1.3)	
8575	683 (2.5)	651 (2.5)	32 (2.4)	
Other	2396 (8.9)	2208 (8.6)	188 (14.1)	
**Grade**				<0.001
I	546 (2.0)	532 (2.1)	14 (1.1)	
II	4585 (17.1)	4368 (17.1)	217 (16.3)	
III	21509 (80.1)	20432 (80.0)	1077 (81.0)	
IV	223 (0.8)	201 (0.8)	22 (1.7)	
**Stage T**				<0.001
I	11371 (42.3)	11239 (44.0)	132 (9.9)	
II	11367 (42.3)	10969 (43.0)	398 (29.9)	
III	2417 (9.0)	2162 (8.5)	255 (19.2)	
IV	1708 (6.4)	1163 (4.6)	545 (41.0)	
**Stage N**				<0.001
0	17268 (64.3)	16998 (66.6)	270 (20.3)	
1	6611 (24.6)	6016 (23.6)	595 (44.7)	
2	1674 (6.2)	1515 (5.9)	159 (12.0)	
3	1310 (4.9)	1004 (3.9)	306 (23.0)	
**Tumor size (cm)**				<0.001
<1.0	3692 (13.7)	3653 (14.3)	39 (2.9)	
1.0–2.0	7657 (28.5)	7533 (29.5)	124 (9.3)	
2.0–5.0	11819 (44.0)	11304 (44.3)	515 (38.7)	
>5.0	3695 (13.8)	3043 (11.9)	652 (49.0)	
**Surgery**				<0.001
No	1724 (6.4)	1018 (4.0)	706 (53.0)	
Yes	25139 (93.6)	24515 (96.0)	624 (46.9)	
**Chemotherapy**				
				0.014
No	6596 (24.6)	6307 (24.7)	289 (21.7)	
Yes	20267 (75.4)	19226 (75.3)	1041 (78.3)	
**Radiotherapy**				<0.001
No	13822 (51.5)	12769 (50.0)	1053 (79.2)	
Yes	13041 (48.5)	12764 (50.0)	277 (20.8)	

8500, Intraductal carcinoma; 8523, Infiltrating duct mixed with other type of carcinoma; 8575, Metaplastic carcinoma.

### Risk factors for distant metastasis of the entire TNBC cohort

All the variables used in chi-square test are also recruited into univariate logistic regression analysis. The univariate logistic model exhibited increased odds of distant metastasis among patients who were of black race (OR = 1.3; 95% CI = 1.2–1.5, *P*<0.001), other histologic type (OR = 1.7; 95% CI = 1.5–2.0, *P*<0.001), grades II–IV, stage T II–IV, stage N1–3, tumor size > 1 cm (all OR > 1, *P*<0.05). Comparatively, those patients who were married (OR = 0.6; 95% CI = 0.5–0.7, *P*<0.001), histologic type 8523 (OR = 0.5; 95% CI = 0.3–0.7, *P*=0.002), surgery (OR = 0.09; 95% CI = 0.07–0.10, *P*<0.001), and radiotherapy (OR = 0.3; 95% CI = 0.2–0.4, *P*<0.001), indicated decreased odds of distant metastasis. More specifically, the multivariate logistic regression analysis revealed an increased risk of distant metastasis among patients with age > 50, stage T III–IV, stage N1-3, tumor size > 5 cm (all OR > 1, *P*<0.05), but a decreased risk of distant metastasis among patients with other race, histologic type 8523, surgery and radiotherapy (all OR < 1, *P*<0.05). Hence age > 50, stage T III–IV, higher stage N, tumor size > 5 cm were independent risk factors for distant metastasis of primary TNBC. The detailed results of logistic regression analysis can be found in Table 2.

**Table 2:** Risk factors associated with distant metastasis of TNBC patients (*n*=26863)

Variables	Univariate logistic model		Multivariate logistic model	
	OR (95% CI)	*P*-value	OR (95% CI)	*P*-value
**Age (years)**				
<35	Reference		Reference	
35–50	0.8 (0.6–1.1)	0.158	1.1 (0.8–1.5)	0.623
50–65	1.1 (0.8–1.4)	0.465	1.7 (1.2–2.3)	0.001
>65	1.1 (0.9–1.5)	0.324	1.6 (1.1–2.2)	0.005
**Race**				
White	Reference		Reference	
Black	1.3 (1.2-1.5)	<0.001	1.0 (0.9–1.2)	0.944
Others	0.9 (0.7–1.1)	0.333	0.7 (0.5–0.9)	0.014
**Marital status**				
Not married	Reference		Reference	
Married	0.6 (0.5–0.7)	<0.001	0.9 (0.8–1.1)	0.085
**Histologic type**				
8500	Reference		Reference	
8523	0.5 (0.3–0.7)	0.002	0.5 (0.3–1.0)	0.036
8575	1.0 (0.7–1.4)	0.939	1.2 (0.8–1.8)	0.383
Other	1.7 (1.5–2.0)	<0.001	1.0 (0.8–1.2)	0.773
**Grade**				
I	Reference			
II	1.9 (1.1–3.3)	0.023	1.1 (0.6–2.2)	0.704
III	2.0 (1.2–3.4)	0.011	1.1 (0.6–2.1)	0.823
IV	4.2 (2.1–8.3)	<0.001	1.3 (0.6–3.1)	0.532
**Stage T**				
I	Reference		Reference	
II	3.1 (2.5–3.8)	<0.001	1.6 (0.9–2.8)	0.077
III	10.0 (8.1–12.5)	<0.001	2.3 (1.4–3.9)	0.001
IV	39.9 (32.7–48.7)	<0.001	6.0 (3.7–9.7)	<0.001
**Stage N**				
0	Reference		Reference	
1	6.2 (5.4–7.2)	<0.001	3.0 (2.6–3.6)	<0.001
2	6.6 (5.4–8.1)	<0.001	3.5 (2.8–4.5)	<0.001
3	19.2 (16.1–22.9)	<0.001	7.8 (6.3–9.7)	<0.001
**Tumor size (cm)**				
<1.0	Reference		Reference	
1.0–2.0	1.5 (1.1–2.2)	0.019	1.2 (0.8–1.8)	0.316
2.0–5.0	4.3 (3.1–5.9)	<0.001	1.3 (0.7–2.4)	0.355
>5.0	20.1 (14.5–27.8)	<0.001	1.9 (1.1–3.3)	0.021
**Surgery**				
No	Reference		Reference	
Yes	0.04 (0.03–0.05)	<0.001	0.09 (0.07–0.10)	<0.001
**Chemotherapy**				
No	Reference			
Yes	1.2 (1.1–1.4)	0.014	1.2 (0.9–1.5)	0.055
**Radiotherapy**				
No	Reference		Reference	
Yes	0.3 (0.2–0.4)	<0.001	0.5 (0.4–0.6)	<0.001

Abbreviation: NI, not included.

8500, Intraductal carcinoma; 8523, Infiltrating duct mixed with other type of carcinoma; 8575, Metaplastic carcinoma.

### Risk factors for bone metastasis of the TNBC patients

In order to characterize which factors would lead to the higher probability of bone metastasis in the TNBC patients, we specifically focused on those patients with bone-only metastasis and excluded 817 patients with other metastasis from the entire cohort. In univariate logistic regression analysis, black race (OR = 1.5; 95% CI = 1.2–2.0, *P*=0.003), other histologic type (OR = 1.9; 95% CI = 1.3–2.6, *P*<0.001), higher stage T and N (OR > 1; *P*<0.001), tumor size > 2 cm (OR > 1; *P*<0.001), were significantly associated with higher risks of bone-only metastasis. The ORs of grade and chemotherapy (*P*>0.05) were insignificant in univariate logistic regression analysis, so they were not enrolled into the subsequent multivariate analysis. After adjusting confounding factors, the multivariate logistic regression model confirmed that clinical stage T>I and N>0 (OR > 1; *P*<0.001) were still significantly associated with higher risks of bone-only metastasis. As a result, higher clinical stage T and stage N were independent risk factors for bone metastasis of primary TNBC. The concrete results of logistic regression analysis for bone metastasis can be seen in Table 3.

**Table 3:** Risk factors associated with bone metastasis of TNBC patients (*n*=26046)

Variables	Univariate logistic model		Multivariate logistic model	
	OR (95% CI)	*P*-value	OR (95% CI)	*P*-value
**Age (years)**				
<35	Reference		Reference	
35–50	0.7 (0.4–1.3)	0.215	1.0 (0.5–1.9)	0.945
50–65	1.1 (0.6–2.0)	0.717	1.8 (0.9–3.2)	0.070
>65	1.1 (0.6–2.0)	0.724	1.6 (0.9–3.0)	0.137
**Race**				
White	Reference		Reference	
Black	1.5 (1.2–2.0)	0.003	1.2 (0.9–1.6)	0.204
Others	0.8 (0.5–1.3)	0.348	0.6 (0.4–1.1)	0.117
**Marital status**				
Not married	Reference		Reference	
Married	0.6 (0.5–0.8)	<0.001	0.9 (0.7–1.3)	0.728
**Histologic type**				
8500	Reference		Reference	
8523	0.4 (0.1–1.3)	0.138	0.5 (0.2–1.7)	0.267
8575	0.8 (0.3–2.0)	0.632	0.9 (0.4–2.4)	0.915
Other	1.9 (1.3–2.6)	<0.001	1.1 (0.8–1.6)	0.655
**Grade**				
I	Reference		NI	
II	1.6 (0.6–4.5)	0.360		
III	1.3 (0.5–3.5)	0.627		
IV	2.6 (0.7–10.6)	0.177		
**Stage T**				
I	Reference		Reference	
II	2.8 (1.8–4.2)	<0.001	2. 9 (1.1–7.4)	0.027
III	9.1 (5.8–14.2)	<0.001	4.4 (1.8–10.5)	0.001
IV	27.6 (18.2–41.9)	<0.001	6.9 (3.1–15.5)	<0.001
**Stage N**				
0	Reference		Reference	
1	6.1 (4.4–8.4)	<0.001	3.1 (2.2–4.3)	<0.001
2	7.3 (4.8–11.2)	<0.001	3.8 (2.4–6.0)	<0.001
3	14.7 (10.0–21.7)	<0.001	5.7 (3.7–8.7)	<0.001
**Tumor size (cm)**				
<1.0	Reference		Reference	
1.0–2.0	1.9 (0.9–4.1)	0.113	1. 7 (0.7–3.7)	0.211
2.0–5.0	4.1 (2.0–8.3)	<0.001	0.9 (0.3–2.7)	0.858
>5.0	17.2 (8.4–35.2)	<0.001	1.2 (0.5–3.2)	0.656
**Surgery**				
No	Reference		Reference	
Yes	0.05 (0.04–0.06)	<0.001	0.1 (0.08–0.14)	<0.001
**Chemotherapy**				
No	Reference		NI	
Yes	1.2 (0.9–1.6)	0.285		
**Radiotherapy**				
No	Reference		Reference	
Yes	0.4 (0.3–0.5)	<0.001	0.8 (0.5–1.1)	0.096

Abbreviation: NI, not included.

8500, Intraductal carcinoma; 8523, Infiltrating duct mixed with other type of carcinoma; 8575, Metaplastic carcinoma.

### The distant metastasis pattern of primary TNBC

In the present study, a total of 1330 cases with distant metastasis were further analyzed. Bone, brain, liver, and lung covered the majority of breast cancer metastasis, so we focused on these four sites. Fifteen possible metastatic forms had been analyzed, including four single metastases and eleven combinative metastasis. Among those TNBC patients, lung-only metastasis was the most frequent (19.6%), bone-only metastasis was the second most frequent (19.4%), while brain-only metastasis occupied least of all (2.9%). As for two metastatic sites, bone+liver accounted for most of those patients (7.4%). As for three metastatic sites, bone+liver+lung occupied most (4.2%). There were 19 cases for four sites metastasis (1.4%). The metastatic pattern of TNBC patients was presented in Table 4.

**Table 4:** The distribution of different distant metastasis (*n*=1330)

Metastatic sites	Patients, number	Percentage (%)
**One site**		
Bone only	258	19.4
Brain only	38	2.9
Liver only	122	9.2
Lung only	261	19.6
**Two sites**		
bone+brain	16	1.2
bone+liver	98	7.4
bone+lung	77	5.8
brain+liver	3	0.2
brain+lung	31	2.3
liver +lung	67	5.0
**Three sites**		
bone+brain+liver	10	0.8
bone+brain+lung	15	1.1
bone+liver+lung	56	4.2
liver+lung+brain	4	0.3
**Four sites**		
bone+liver+lung+brain	19	1.4

### Survival analysis

To better understand the relationship between distant metastasis and follow-up time, we further analyzed the influence of each distant metastasis on patients’ survival. Of the 26863 patients finally recruited, 4433 patients were dead at the end of the last follow-up. Moreover, 3526 patients died from breast cancer specifically. The Kaplan–Meier plots displayed that TNBC patients with brain metastasis had the worst survival in both BCSS and OS, though the survival difference was not statistically significant (*P*>0.05, respectively). As a result, each distant metastasis may exert poor survival for the TNBC patients. The survival curves of BCSS and OS are exhibited in Figure 1.

**Figure 1:** Kaplan–Meier estimates of BCSS and OS in each distant metastasis (**A**) BCSS for only one site metastasis: χ^2^ = 7.346, *P*=0.062. (**B**) OS for only one site metastasis: χ^2^ = 6.337, *P*=0.096.

In order to distinguish bone metastasis alone from bone combined with other organ metastasis, we further analyzed the survival difference between bone-only metastasis and bone with other sites metastasis. The Kaplan–Meier plots indicated that bone combined with other metastasis exerted significantly worse survival for the TNBC patients. The survival curves of BCSS for these patients are available in Figure 2.

**Figure 2:** Survival curves of bone metastasis Kaplan–Meier estimates of BCSS for TNBC patients with bone-only metastasis and bone with other organ metastasis: χ^2^ = 42.98, *P*<0.001.

Specifically, the median BCSS of the entire cohort was 13 months, the median OS was also 13 months. TNBC patients with either lung or liver metastasis experienced the longest median BCSS (15 months), while those with bone-only metastasis had relatively shorter survival (14 months), but the survival difference was not significant (Figure 1). Bone combined with other organ metastasis engendered worse survival than bone metastasis alone (median BCSS: 8 vs 14 months). By contrast, the patients with brain-only metastasis had the shortest median survival (5 months). Consequently, TNBC patients with either bone or visceral metastasis had poor survival.

The patients with brain metastasis have the worst survival. The number and median survival of those patients with different metastasis are listed in Table 5.

**Table 5:** The median survival of TNBC patients with different metastasis (*n*=1330)

Metastatic site	Patients, number	Median BCSS	Median OS
		95% CI, months	95% CI, months
Overall	1330	13 (12.2–13.8)	13 (12.2–13.8)
Bone only	258	14 (12.4–15.6)	13 (11.5–14.5)
Brain only	38	5 (2.6–7.4)	5 (2.6–7.4)
Liver only	122	15 (12.8–17.2)	14 (12.2–15.8)
Lung only	261	15 (12.2–17.8)	15 (12.5–17.5)
Bone+other	291	8 (6.3–9.7)	8 (6.3–9.7)

## Discussion

Multiple factors, such as age at diagnosis, tumor site, laterality, stage, lymph node involvement, ER/PR and HER2 status etc., have been linked to an elevated risk of developing distant metastasis in breast cancer [6]. Nevertheless, few studies have specifically focused on the risk factors for distant metastasis of patients with primary TNBC. In the present study, we extracted a large patient cohort from the SEER database to analyze several potential risk factors for distant metastasis of TNBC, including patients’ demographics, tumor features and treatment. According to the descriptive statistical analysis, univariate and multivariate logistic regression analyses, we have found that age > 50, clinical stage T III-IV, higher stage N, tumor size > 5 cm were independent risk factors for distant metastasis of primary TNBC. Moreover, we also investigated different distant metastasis pattern and survival of the patients. The overall results indicated that lung metastasis is the most frequent while brain metastasis is the least frequent in TNBC. The patients with brain metastasis had the worst survival, though the OS difference among the four metastatic sites was not significant. Generally, TNBC patients with each distant metastasis had poor survival.

Age is a very important prognostic factor of breast cancer. Several previous reports showed that younger age was associated with distant metastasis and poor prognosis. A recent study indicated that patients ≤35 had 2.51-times greater risk of recurrence-free survival, and 2.60-times greater risk of distant recurrence compared with the patients >50 years old. However, this study did not specifically focus TNBC, and the sample size of TNBC was only 143 [7]. Another study recruited 1930 patients with TNBC, 15% were <40 and 85% were ≥40 years of age at diagnosis. At a median follow-up of 74 months, there was no significant difference in local recurrence (LR) or disease-free survival (DFS) between patients <40 and ≥40 years old. The conclusion was ‘Young age at diagnosis is not an independent risk factor for LR or DR in patients with TNBC’ [8]. Furthermore, another report has compared the clinical pathological characteristics of <65 and ≥65 years old TNBC patients. The results showed that distant visceral metastases occurred significantly more often than bone metastases in both age groups. LR, bone and secondary lymph node metastases were significantly more frequent in younger patients [9]. Comparatively, our results indicated that TNBC patients with age > 50 were independent risk factors for distant metastasis. The possible reasons for these disparities may be as follows. Our study specifically concentrated on TNBC rather than other breast cancer subtypes. We also enrolled a much larger population of TNBC patients, so the power of analysis in our study seemed more convincing.

The present study identified clinical stages T and N were independent risk factors for distant metastasis of primary TNBC. Several previous reports have indicated a relation of increasing lymph node involvement with poorer prognosis of TNBC patients. A recent study revealed that 5-year progression-free survival (PFS) was significantly worse in patients with FNAB(+) IMN metastasis. The FNAB(+) IMN patients showed worse distant metastasis and regional recurrence-free survival [10]. Furthermore, another study has evaluated the prognostic value of the lymph node ratio (LNR) in patients with axillary lymph node-positive TNBC. It revealed that the LNR was an independent predictor of OS in high-risk patients. Considering the heterogeneity of TNBC, the LNR exhibits potential as an additional prognostic factor for TNBC patients with positive lymph node involvement [11]. In our study, we have also found that higher clinical N-stage is associated with increased ORs of distant metastasis. Hence routine evaluation of the internal mammary and axillary lymph node should be considered for early detection of TNBC metastasis.

Some scholars have reported that tumor sizes < 1 cm are independent risk factors for TNBC. The tumors ≤ 1 cm are difficult to treat as recurrence rates are tough to estimate. A recent report has evaluated outcomes of patients who had tumors ≤ 1 cm, node negative and investigated their recurrence by both underlying triple receptor subtypes and by age. The results presented that women with small tumors often had aggressive underlying biology and unfavorable prognosis [7].

On the other hand, prior research on TNBC also reported that larger tumors were associated with worse survival [12]. Lymph nodal metastasis was more frequent in TNBC with large tumor size, which was also associated with late stage at presentation [13]. Our study determined that tumor size > 5 cm was an independent risk factor for distant metastasis of primary TNBC. The elevated likelihood of distant metastasis from large tumor size can be possibly interpreted by the contribution of increased time to presentation since larger tumors require more time to grow [14]. In addition, it is difficult to perform surgical resection and procure adequate margins for larger tumors. The risk of distant metastasis increases as residual cancer cells continue to divide untreated over time [15]. Thus great concern should be taken on large tumor size, in order to identify high-risk groups of TNBC patients with distant metastasis.

As far as the distant metastasis pattern of TNBC is concerned, previous study reported a higher incidence of visceral metastasis while less frequent in bone metastasis [16]. Consistently, our study revealed that lung-only metastasis (19.6%) was the most frequent while bone-only metastasis was relatively lower (19.4%) among single organ metastasis. The specific metastatic organ involved can predict prognosis of the patients [17]. Some studies revealed that breast cancer with bone metastasis alone was associated with better prognosis, whereas those with bone and visceral pattern had the worse prognosis [18]. Concordantly, our study also indicated that TNBC patients with bone-only metastasis had better survival than bone combined with other metastasis. Furthermore, the prognosis of bone-only metastasis is not significantly different from lung- or liver-only metastasis. The higher percentage of patients with bone-only metastases could be partially explained by the growing number of TNBC patients with higher clinical stage. We also found that higher clinical stage T and stage N were independent risk factors for bone metastasis of primary TNBC. As a matter of fact, knowledge of the risk factors for distant metastasis of TNBC may become useful for evaluating the prognosis of the patients.

Several limitations should be considered in our study. First, this is a retrospective study from SEER database rather than a prospective cohort study, so the inherent selection biases may undermine the external validity of the present study. Second, the information about TNBC recurrence and subsequent sites of metastasis are not available in the SEER database, so we could not evaluate patients who developed distant metastasis later in their disease course. Third, we did not analyze other potential risk factors such as smoking status and comorbidities. The reason was that the SEER database did not provide any data on these variables.

## Conclusion

In summary, age > 50, higher stage T and N, and larger tumor size were independently associated with higher risks of distant metastasis in primary TNBC. The risk factors characterized in the present study may help clinicians in counseling patients about the likelihood of distant metastasis at initial diagnosis. Improving our understanding of the risk factors for distant metastasis of TNBC may also contribute to the current individualized treatment for these patients.

## Abbreviations

AJCC: American Joint Committee on Cancer
BCSS: breast cancer-specific survival
CI: confidence interval
ER: estrogen receptor
FNAB: fine needle aspiration biopsy
HER2: human epidermal growth factor receptor 2
IMN: internal mammary lymph node
LNR: lymph node ratio
LR: local recurrence
OR: odds ratio
OS: overall survival
PR: progesterone receptor
SEER: Surveillance, Epidemiology, and End Results
TNBC: triple-negative breast cancer
